# Resin Composite Materials for Chairside CAD/CAM Restorations: A Comparison of Selected Mechanical Properties

**DOI:** 10.1155/2021/8828954

**Published:** 2021-04-28

**Authors:** Wojciech Grzebieluch, Marcin Mikulewicz, Urszula Kaczmarek

**Affiliations:** ^1^Laboratory for Digital Dentistry, Department of Conservative Dentistry witch Endodontics, Wroclaw Medical University, Krakowska 26, Wrocław 50-425, Poland; ^2^Department of Dentofacial Orthopeadics and Orthodontics, Division of Facial Abnormalities, Wroclaw Medical University, Krakowska 26, Wrocław 50-425, Poland; ^3^Department of Conservative Dentistry witch Endodontics, Wroclaw Medical University, Krakowska 26, Wrocław 50-425, Poland

## Abstract

**Objective:**

The aim was to evaluate the flexural strength, flexural modulus, microhardness, Weibull modulus, and characteristic strength of six resin composite blocks (Grandio Blocs-GR, Tetric CAD-TE, Brilliant Crios-CR, Katana Avencia-AV, Cerasmart-CS, and Shofu Block HC-HC).

**Methods:**

Flexural strength and flexural modulus were measured using a three-point bending test and microhardness using the Vickers method. Weibull analysis was also performed.

**Results:**

The materials showed flexural strength ranging from 120.38 (HC) to 186.02 MPa (GR), flexural modulus from 8.26 (HC) to 16.95 GPa (GR), and microhardness from 70.85 (AV) to 140.43 (GR). Weibull modulus and characteristic strength ranged from 16.35 (CS) to 34.98 (TE) and from 123.45 MPa (HC) to 190.3 MPa (GR), respectively.

**Conclusions:**

GR, TE, and CR presented significantly higher flexural strength, modulus, Weibull modulus, and characteristic strength than the others.

## 1. Introduction

During the last years, a significant increase in the use of computer-aided design and computer-aided manufacturing (CAD/CAM) of indirect dental restorations was noticed [1–3].

It resulted from the progress in intraoral imaging, manufacturing technology, hardware development, software, and monolithic materials referred to as blocks suitable for CAD/CAM transfer. Digital systems provide an opportunity to fabricate esthetic fixed restoration within one visit due to the elimination of a number of steps typical of the traditional technique. The rapid fabrication at the chairside of tooth-colored restorations has been obtained by optical impression-taking, designing, and machining. A wide diversity of materials is used for CAD/CAM restorations. These materials are manufactured with the guarantee of desired chemical and physical properties and have superior mechanical strength compared to their conventionally manufactured equivalents [4].

The CAD/CAM materials can be classified as metal, ceramics, resin (polymethyl methacrylate-PMMA, resin composite, nanoceramics), and polymer-infiltrated-ceramic-network material (PICN) [5]. Two types of materials are used currently for aesthetic chairside indirect restorations: glass ceramics/ceramics and resin composites.

CAD/CAM resin composites represent a relatively new group of materials, many of them are relatively new and there is a lack of scientific literature data regarding their mechanical properties. The differences between resin composites and ceramic materials are widely known and resulting from their composition and structure, which influence their mechanical properties. Glass-ceramics/ceramics materials display considerably higher values of the flexural modulus (*E*_*f*_) and Vickers hardness than resin composites (≥60 GPa, >4 GPa versus 9–20 GPa, 0.4 GPa, respectively). Despite such significant differences, both types of materials are widely and successfully used in restorative dentistry. Resin composite consists of ceramic powders (or ceramic network) and resins are easier to mill and repair intraorally [6–8].

Available long-term clinical studies have proven the durability of CAD/CAM CEREC® (Sirona Dental, Bensheim, Germany) ceramic restorations with a survival rate of 97% within 5 years, 95.5% within 9 years, and 88.7% within 17 years [9–12]. Unfortunately, due to the relatively short availability on the market, there is no long-term clinical trial on CAD/CAM resin composite blocks. Due to the wide range of composite materials for milling, a prediction of clinical success of the chosen material, in practice, is based mainly on their aesthetic properties and less on the mechanical ones that should be similar to the tooth structure. Most of the data is provided by the manufacturers. However, we can find a significant discrepancy in the results, difficult to be explained only by the methodology differences [6, 13, 14].

The aim of the study was to compare flexural strength, flexural modulus, hardness, and probability of failure of 6 commercially available resin composite CAD/CAM materials.

## 2. Materials and Methods

### 2.1. Study Design

The comparison of flexural strength, flexural modulus, microhardness, Weibull modulus, and characteristic strength of six composite materials for chairside CAD/CAM system was conducted. The tested composite CAD/CAM blocks were Grandio blocs® (VOCO, Cuxhaven, Germany), Tetric CAD® (Ivoclar Vivaden, Schaan, Liechtenstein), Brilliant Crios® (Coltene/Whaledent A.G. Altstatten, Switzerland), Katana Avencia Block® (Kuray Noritake Dental, Tokyo, Japan), Cerasmart® (GC Dental Product Europe, Leuven, Belgium), and Shofu Block HC® (Shofu Inc., Kyoto, Japan), their composition according to literature is placed in Table 1 [15–20].

### 2.2. Samples Fabrication

The CAD/CAM blocks were cut with a low speed water-cooled diamond saw Miracut 151 (Metcon, Bursa, Turkey) to obtain sixty bar-shaped specimens, ten for each material. Specimens were finished by a glass grinder (JZO, Jelenia Gora, Poland) with wet silicon carbide (initially 240 ISO/FEPA, average grain size 68 *μ*m and finally 400 ISO/FEPA, average grain size 35 *μ*m) until dimensions of 15 mm long, 4 mm wide, and 1.5 mm thick were reached according to ISO 6872:2015 (accuracy 0.01 mm) [21]. The samples were stored dry at room temperature. Sample preparation according to ISO 4049 was not possible due to the size of the material blocks [22].

### 2.3. Methods

Flexural properties were measured using a three-point bending test that was conducted with a support span of 12 mm and a speed of 1 mm/min using a universal testing machine LabTest 5.030S LaborTech® (LaborTech Opava, Czech Republic) equipped with Test&Motion® (LaborTech Opava, Czech Republic) software (in accordance with the ISO 6872:2015) [21].

The flexural strength (*σ*_*f*_) was calculated from the three-point bending results using the following formula:

(1) $$\begin{array}{c} \sigma_{f}=\frac{3Fl}{2wh^{2}}, \end{array}$$

where *F* is the maximum load during the flexural test, *l* the roller span (12 mm), *w* the width (4 mm), and *h* the height (2 mm) of the bar.

The flexural modulus (*E*_*f*_) was calculated from the three-point bending results using the following formula:

(2) $$\begin{array}{c} E_{f}=\frac{Fl^{3}}{4wh^{3}d}, \end{array}$$

where *F* is the load, *l* the roller span (12 mm), *w* the width (4 mm) and *h* the height (2 mm) of the bar, *d* is the deflection corresponding to load *F*.

The microhardness was measured by means of a Vickers intender tester (Shimadzu HMV-2T, Shimadzu Corp. Kyoto, Japan) with a load of 980.7 mN (HV 0.1) and dwell time of 10s. Five indentations were applied in a random location for each specimen. Then, the machine automatically calculated the hardness value as HV 01. Before the measurement, surfaces of the samples were sequentially polished with composite rubbers HiLusterPlus® Polishing System (Kerr Corp., Orange, CA, USA). The microhardness measurements were carried out on the same samples that were used in a three-point bending test.

### 2.4. Statistical Analysis

The obtained data were tested using one-way ANOVA analysis for homogeneity of variance (*p* < 0.05), following multiple comparisons post hoc Tukey's test using Statistica 13 PL software (StatSoft Poland). The significance level was set at *p* ≤ 0.05. Weibull statistics were also carried out to obtain the shape and scale parameters. Weibull modulus (*m*) and probability of failure (*P*_*f*_) were calculated using the following equation:

(3) $$\begin{array}{c} P_{f}=1-\exp\left[-N\cdot {\left(\frac{\sigma }{\sigma_{0}}\right)}^{m}\right], \end{array}$$

where *m* is Weibull modulus, *σ*_0_ is Weibull characteristic strength, and *σ* is flexural strength.

## 3. Results

Mean flexural strength, flexural modulus, and microhardness for all tested materials are shown in Table 2 and Figures 1–3. A statistically significant difference between means of all studied parameters was found.

The values of flexural strength ranged from 120.38 (SD 6.54) MPa for HC to 186.02 (SD 10.49) MPa for GR. Flexural strength of GR was significantly higher in comparison to the other tested materials (*p* < 0.001) and was also significantly higher for TE and CR compared to AV and CS, and for TE, CR, AV, and CS compared to HC. No significant differences between the pairs CR-TE and AV-CS were found. Flexural strength ranged in the decreasing order as follows: GR > TE > CR > AV > CS > HC.

The flexural modulus values ranged from 8.26 (SD 0.55) GPa for HC to 16.95 (SD 0.50) GPa for GR. The flexural modulus of GR was significantly higher in comparison to the other tested materials and was also higher for TE and CR compared to AV, CS and HC. The values of flexural modulus changed in the descending order as follows: GR > CR > TE > CS > AV > HC.

The values of microhardness ranged from 70.85 (SD 1.62) for AV to 140.43 (SD 5.47) for GR. The microhardness of GR was significantly higher compared to the other tested materials. Similar values for TE and CS as well as for CR and HC were found. The microhardness values in the diminishing order were as follows: GR > HC > CR > TE > CS > AV.

Calculated Weibull modulus (*m*) ranged from 16.35 for CS to 34.89 for TE. The ranking of the Weibull modulus was as follows CS > HC > AV > GR > CR > TE. Weibull survival curves of the flexural strength, showing a probability of failure (*P*_*f*_) at any stress level, are shown in Figure 4. Weibull characteristic strength (*σ*_0_) ranged from 123.45 for HC to 190.30 for GR (Table 2). The values of Weibull characteristic strength (*σ*_0_) in the diminishing order were as follows: GR > CR > TE > AV > CS > HC.

## 4. Discussion

Mechanical properties of dental materials are assessed based on the results of in vitro testing. The characteristics of dental materials in laboratory conditions can predict clinical performance to some extent although an imitation of an oral environment is difficult to be reconstructed in vitro. International Standard Organization elaborated protocols, standardized testing methods, and the required qualities allow for comparisons of dental restorative material properties. The test results performed according to the standard procedures can eliminate the unfounded claims of manufacturers regarding material superiority and predict the success of the dental material in clinical conditions [23].

Dental restorative materials, besides fulfillment of the aesthetic demands, ought to withstand the biomechanical forces placed upon them during function. Because dental restorations are static entities, all mechanical properties of the restorative materials are measured regarding their resistance to deformation or fracture under the applied load [23].

The forces acting upon material are mainly tensile, compressive, shearing, and torsional. Additionally, bending forces being a compilation of tension, compression, and shear forces are subjected intraorally. Despite the common failure of dental materials caused by tensile stress, any force applied to a restoration is probably a combination of tensile, compressive, and shear forces. Consequently, flexural strength, tested with the use of a three-point bending test, reflects compressive and shear stresses in the same sample, and it is the best way to mimic stresses which are applied on the dental materials in oral condition [24–26].

The flexural strength presents the greatest stress experienced by the material at the time of failure. Therefore, a high value of *σ*_*f*_ is a required property for the indirect restoration materials to withstand the forces of mastication without fracture.

The tested materials are designed for permanent indirect single-tooth restorations such as inlays/onlays, veneers, partial crowns, or full crowns. Therefore, they should have mechanical properties resembling those of hard dental tissues. In our study, the measured flexural strength after dry storage of the samples differed from 120.38 to 186.02 MPa (about 65%). However, the obtained values were comparable with those of the dentine, which varied from 109 ± 10 to 212.9 ± 41.9 MPa [27, 28]. Of the studied CAD/CAM materials, GR, being the most filled composite material in this comparison, revealed the highest value of flexural strength compared to other materials. However, it was much lower than the biaxial flexural strength given by the manufacturer (186.02 MPa vs. 333 MPa, respectively) [16]. The difference seems to be too large to be explained by the use of a different measurement method [29]. TE and CR revealed slightly lower strength, around 170 MPa. TE showed much lower than the biaxial flexural strength given by the manufacturer (170.65 MPa vs. 273.79 MPa, respectively) [17]. CR had some lower flexural strength in comparison to the one found in the literature recorded after 24 h water storage (170.46 vs. 198 MPa) [30]. CS turned out also to have a lower value of flexural strength than the manufacturer's data and the results of other studies, regardless of the material storage [20, 25, 31–34]. Similarly, HC revealed lower flexural strength than the manufacturer's data and the results of other studies obtained after dry storage and similar to data obtained after thermocycling and water storage [20, 30]. GR, TE, and CR presented significantly higher flexural strength than the other materials, whereas the CS, having a similar filler content to TE and CR, showed significantly lower strength. The recorded flexural strength values, lower than those reported by other authors and manufacturers, may be the result of the difference in applied methodology (e.g., the roughness of the sample surface, the roller span, and geometry of the samples) and also the material manufacturing process deviations [20, 25, 30, 31, 33, 34].

The flexural strength is the important parameter that determines the material properties but does not determine how the material will be deformed during loading. Therefore, for a better understanding of material behavior, it is necessary to determine elastic properties by measuring the flexural modulus. The 3-point bend test allows calculating simultaneously the flexural strength and the flexural modulus *E*_*f*_. The flexural modulus is called “modulus of elasticity in bending,” or “modulus of elasticity” or “elastic modulus,” or simply “modulus” is represented by the slope of the stress-strain curve obtained during the first or initial step of the 3-point bend test and determines the stiffness [21, 25, 26].

*E* moduli of the dental hard tissues based on the literature range from 74 to 130 GPa for the human enamel and from 17.7 to 29.8 GPa for the dentine [35–38]. Comparison of these parameters reveals a significant difference between enamel and dentine. Mechanical properties of the tissues, including *E* modulus, change within a tooth structure depending on the location and depend on many factors, e.g., mineralization, tubule density, and orientation [35, 39].

The obtained results showed that the tested materials, stored in dry conditions, presented much smaller values of elastic modulus compared to the enamel. Only one of the tested materials-GR revealed the flexural modulus value close to the dentine ones. The GR flexural modulus was highest and nearly 2-fold higher than the values recorded for AV, CS and HC. CR and TE presented lower flexural modulus than GR, but significantly higher compared to the values recorded for AV, CS, and HC. The flexural modulus values recorded for GR, CR, and HC were similar to values obtained in different research papers [18, 20, 25, 30]. The HC revealed a lower value of flexural modulus than the one given by Lauvahutaton et al. in dry conditions [20]. The CS flexural modulus value obtained in this study was lower compared to the study by Lauvahutaton et al. [20] and Lawson et al. [32] and higher than reported by Awada and Nathanson [25].

Resin composites tested in this study are made of resin bonded filler which results in much lower *E* module values than those of enamel. It is worth mentioning, a new type of material-polymer infiltrated ceramic-network (PICN) is manufactured not by polymerization of the resin mixed with powder but by resin infiltration of a porous sintered solid ceramic block. As a result of this process, a composite with *E* modulus of 27.26 to 37.95 GPa is obtained [5, 40, 41]. However, this material has lower flexural strength values than most CAD/CAM resin composites reviewed in this study. It exceeds only the flexural strength of HC [42].

Materials with low *E* modulus values transfer more loads inside the tooth structures than stiffer ceramic materials [43]. Despite them, the clinical results of resin composites do not differ from gold cast restorations [44].

The surface hardness of a dental material can be considered as a predictor of the wear resistance of a material [35, 45]. However, the lower hardness of the CAD/CAM materials contributes to their milling susceptibility [6].

Microhardness testing (Vickers) revealed that GR, containing 86% filler by weight, was the hardest among the studied CAD/CAM materials, nearly 2-fold harder than the others. The obtained result was slightly lower compared to the manufacturer's data [16] (140.43 vs. 154.6) and higher compared to the data obtained by Alamoush et al. [15], (140.43 vs. 121.8). Similarly, CS microhardness was higher compared to Lauvahutaton et al. [20], Lawson et al. [32], and Kamonwanon et al. [46]. Microhardness values for HC were higher than the value contained in the independent data and that of the manufacturer's [20, 46]. Kamonwanon et al. [46] found lower hardness value (almost half) for CS, AV, and HC than our results and also lower than those obtained by Alamoush et al. [15], Lauvahutaton et al. [20], and Lawson et al. [32]. The enamel hardness ranges from 270 to 360 and the dentine's from 50 to 62.3 [15, 47]. Our data showed that the hardness of all the tested materials was higher than the dentine's but much lower than the enamel's one. When comparing the microhardness of the resin composite materials, we should also notice that hardness is not a predictor of material wear. The resin composite material wear will not only be the result of friction but also occurs due to chemical degradation caused by an aggressive oral cavity environment [48, 49].

Nowadays, researchers utilize Weibull statistics which is based on “weakest link theory” and allows to estimate the probability of material failure [50–52]. Weibull modulus (*m*) has an important practical indication because a higher *m* value means smaller deviations of flexural strength and indicates better homogeneity of the material. For this reason, materials with higher *m* value are preferable, even in association with slightly lower flexural strength [50–52]. Determining the probability of failure at any possible stress level allows to evaluate the reliability of materials and to estimate the dependability of the tested materials as a load function [53]. Weibull's characteristic strength value estimates that the probability of failure equals 63.2% (*p*_*f*_=63.2%). TE showed the highest *m* value (34.89) at *σ*_0_ of 173.26 MPa, while GR, a material with the highest *σ*_0_ of 190.30 MPa, showed *m* value of 25.72. The *m* and *σ*_0_ values of GR, TE, and CR are higher than recorded for CS (lowest m) and HC (lowest *σ*_0_). Stawarczyk et al. [34] reported lower Weibull modulus and higher characteristic strength values for CS and HC. The difference may be explained in sample surface roughness. Mentioned above authors polished samples up to P4000 (average grain size 2.5 *μ*m) vs. P400 (present study-average grain size 35 *μ*m). However, it should be remembered that the milling machine processes the material with a diamond drills and the obtained surface is affected by the milling process and rough. [54] During clinical procedure, the internal surface of resin composites is usually sandblasted before adhesive cementation (50 *μ*m AlO_2_) and only the external surface is polished.

## 5. Conclusion

Within the limitation of this *in vitro* study, it can be concluded that flexural strength, flexural modulus, and Vickers hardness of the tested materials presented significant differences.

Therefore, clinicians are advised to take into consideration these differences when planning teeth indirect restoration using these materials.

GR, TE, and CR presented significantly higher flexural strength, flexural modulus, Weibull modulus, and Weibull characteristic strength than the others.

There is a need to develop restoration materials (method) in terms of stress-strain behavior more similar to the natural tooth structure.*σ*_*f*_: flexural strength; *E*_*f*_: flexural modulus; HV01: Vickers microhardness; *m*: Weibull modulus; and *σ*_0_: Weibull characteristic strength. Materials with the same letter within a column are not significantly different (*p* > 0.05). Mean values (*n* = 10) and standard deviations in parentheses. *x̅*: mean; SD: standard deviation.

## Figures and Tables

**Figure 1:** Flexural strength of the testing materials.

**Figure 2:** Flexural modulus of the testing materials.

**Figure 3:** Microhardness of the testing materials.

**Figure 4:** Weibull survival curves of the flexural strength of the testing materials.

**Table 1:** Machinable materials used in the study.

Brand	Abr.	Manufacturer	Composition	Lot no.	Shade	Block size
Grandio blocs	GR	VOCO, Cuxhaven, Germany	86 wt % nanohybride fillers, 14% UDMA + DMA [15, 16]	1711521	A2 HT	C 14L
Tetric CAD	TE	Ivoclar vivaden, Schaan, Liechtenstein	Dimethacrylates 28.4 wt%: Bis-GMA, Bis-EMA, TEGDMA, UDMA; fillers: 71, 1 wt%, barium glass (<1 um), silicon dioxide (<20 nm) [17]	35470	3M2 HT	14
Brilliant crios	CR	Coltene/Whaledent A.G. Altstatten, Switzerland	Resin matrix cross-linked methacrylate, 70.7 wt % barium glass (<1 *μ*m), amorphous silica (<20 nm) [15, 18]	H22667	A2 LT	C 14
Katana avencia block	AV	Kuray Noritake dental, Tokyo, Japan	UDMA, TEGDMA with 62 wt % aluminum filler (20 nm), silica filler (40 nm) [19]	000318	A2LT	12
Cerasmart	CS	GC dental product Europe, Leuven, Belgium	BisMEPP, UDMA, DMA with 71% wt% silica (20 nm) and barium glass (300 nm) [15, 19]	37690	A3 C	14
Shofu block HC	HC	Shofu inc., Kyoto, Japan	UDMA, TEGMA, 61 wt% silica powder, micro fumed silica, zirconium silicate [15, 19]	071601	A2 LT	14

UMDA: urethane dimethacrylate; TEGDMA: triethylene glycol dimethacrylate; Bis-GMA: bisphenol A diglycidylether methacrylate; Bis-EMA: ethoxylate bisphenol-A dimethacrylate; DMA: dimethacrylate; Bis-MEEP: 2,2-Bis(4-methacryloxypolyethoxyphenyl) propane; EDMA: ethyleneglycoldimethacrylate; DMA: dimethacrylate.

**Table 2:** Mechanical properties of the testing materials.

Material	*σ*_*f*_ (MPa)	*E*_*f*_ (GPa)	HV01	*m*	*σ*_0_ (MPa)
	*x̅* (SD)	*x̅* (SD)	*x̅* (SD)		
GR	186.02 (10.49) A	16.95 (0.50) A	140.43 (5.47) A	25.72	190.30
TE	170.65 (5.61) B	10.56 (0.19) B	74.88 (2.82) BC	34.89	173.26
CR	170.46 (8.89) B	11.14 (0.16) C	75.40 (2.18) B	27.18	174.16
AV	142.79 (6.56) C	8.39 (0.13) D	70.85 (1.62) C	22.92	145.90
CS	136.27 (9.40) C	8.45 (0.20) D	71.13 (0.92) BC	16.35	140.50
HC	120.38 (6.54) D	8.26 (0.55) D	77.84 (5.11) B	19.62	123.45
*p* value ^*∗*^	**p** < 0.001	**p** < 0.001	**p** < 0.001	—	—

## Data Availability

Data are available upon request.
